# Analysis on the Influence of Table Tennis Elective Course on College Students' Health

**DOI:** 10.1155/2022/8392683

**Published:** 2022-01-17

**Authors:** Ke Zhu, Lina Xu

**Affiliations:** Beijing Sport University, Beijing 100084, China

## Abstract

College physical education elective course is the last physical education course for college students. It also plays an irreplaceable positive role in the formation of College Students' lifelong physical education. Table tennis, as China's national ball, is of great significance to enhance the physique of elective courses. As an elective course of college physical education, table tennis is widely loved by college students. It is a very popular course in college physical education elective courses. This paper discusses the influence of table tennis on health. This paper puts forward the reform scheme of teaching plan design of table tennis elective course in colleges and universities, which has a certain reference value for the development of College Physical Education in China.

## 1. Introduction

In recent years, with the deepening of the reform of physical education curriculum in Chinese universities, the traditional teaching method has been broken. Now, college students can choose the sports they want to learn according to their interests and specialties through elective physical education courses [1]. Elective course is the future and hope of national rejuvenation; their healthy growth is directly related to the prosperity of the country. Since the finding of the People's Republic of China, the party and the government have attached great importance to the health of elective courses, especially for physical education in primary and secondary schools and colleges and universities [2]. Due to the one-sided pursuit of enrollment rate by the society and schools, students' schoolwork burden is too heavy. The serious lack of rest and exercise time and sports facilities and conditions lead to students' physical education and sports activities difficult to guarantee [3]. Table tennis, as the national sport of China, is of great significance to enhance the physique of elective courses. Table tennis is characterized by small ball, fast speed, many changes, strong interest, simple equipment required for the project, less investment, and not limited by age, gender, and physical conditions, so it is easy to be accepted by the public [4].

In today's table tennis teaching, it is necessary to explore new teaching methods and methods. As the last stage of college students' career, physical education elective course plays an important role in the mastery of college students' physical skills, the improvement of physical exercise ability, and the formation of lifelong sports consciousness [5]. Table tennis is China's “national ball,” which has a great influence in the elective group and is also a favorite sport in the elective [6]. In this context, school physical educators should attach great importance to the promotion of table tennis on the healthy development of elective courses and scientifically organize and carry out table tennis training activities of elective courses [7]. It is an indisputable fact that the elective course is at a low level of health. Only when we face this problem squarely can we find a way to solve it. Effective teaching methods and methods not only enable students to master table tennis technology but also guide students to establish the awareness and habit of lifelong physical exercise, so as to improve the physical health level of college students and so as to achieve the purpose of strengthening physique and improving health advocated by the state [8].

This paper is a comprehensive narrative article, which makes a comprehensive discussion on the teaching of table tennis in colleges and universities. This paper not only discusses the impact of table tennis on health but also puts forward the reform scheme of teaching plan design of table tennis elective course in colleges and universities, which has a certain reference value for the development of College Physical Education in China.

## 2. The Influence of Table Tennis on Physical Health

Table tennis, as a sport, has a long history of development in China, and its overall technical level is in the leading position in the world. It not only has won many honors for China in the world's major sports events but also become an important bridge for China's foreign exchanges. With the promotion of the national movement, colleges and universities, as the cradle of cultivating talents, have gathered a large number of vigorous young people. Therefore, we should give full play to the role of physical education so that students learn sports knowledge and, at the same time, exercise and cultivate sports hobbies. Today's students with the improvement of living standards, the popularity of table tennis, from the students themselves, some have a very high level of technology. The elective course of table tennis requires the coordinated movement of multiple parts of the whole body. Whether it is the simple moving pace or the complex hanging ball and rubbing ball technology, it will affect the young people's body in varying degrees. In terms of physiological function, table tennis emphasizes the strong correlation between brain and body movements.

Table tennis is a favorite sport in many elective courses. The huge audience provides good conditions for schools to carry out table tennis education and improve the health level of elective courses. It can effectively improve the level of health education to carry out table tennis elective courses in schools. In this study, the main indexes of students' physical health in a domestic university in recent three years were sampled and measured. In Table 1, the data analysis of physical health status of students in our school in recent three years is shown.

Table tennis elective course, from its own point of view, is a movement with higher requirements for sensitivity and speed, but the requirement for the amount of exercise is relatively small. Therefore, the application of a wide range of groups is a suitable for contemporary college students to carry out sports activities. At the same time, table tennis is more strict in technical essentials, and every skill training and cultivation should be completed through continuous practice and consolidation, which play an immeasurably important role in cultivating students' patience and concentration ability. Although table tennis is called national ball, it has the characteristics of small range of motion and weak antagonism compared with basketball and football. However, because of its high requirements for hardware facilities, great changes have taken place from the initial outdoor cement ball table to the later indoor movable ball table. Whether it is a regular competitive training course or a routine competitive training course, it can improve the confidence of winning and losing. As far as the current situation is concerned, colleges and universities basically take reducing expenditure as the prerequisite for running a school, which cannot meet the basic needs of teachers. Therefore, teachers are greatly restricted in thought, spirit, and action.

The rhythm of table tennis is fast, and it is often in a flash to seize the opportunity to win. Therefore, taking an active part in table tennis can effectively enhance the function of the nervous system. In addition, table tennis can also enhance the functions of the blood circulation system and the respiratory system. In terms of physical fitness, table tennis requires athletes to have strong upper limb strength and lower limb strength. Therefore, taking an active part in table tennis can effectively improve the quality of strength element. According to the principle of students' subjectivity, the main body of table tennis course learning is students, so teachers are required to make the training plan of elective courses according to the overall physical quality of students. Hierarchical teaching needs a distinction according to the level of students' table tennis skills to carry out teaching, which is bound to need the support of school hours and the provision of venues. That is to say, in the past, teachers were taught in one class, but now they need to be divided into ordinary classes and improved classes, which will virtually increase the workload of teachers, so the school has to pay teachers accordingly. The contents of table tennis techniques and tactics are rich. If the elective course wants to make a big show in table tennis, it needs long-term training. In the process of training, the elective course needs to overcome the physical pain and psychological pressure. From this point of view, table tennis can effectively cultivate the strong will quality of elective courses.

## 3. Reform of Teaching Plan Design of Table Tennis Elective Course in Colleges and Universities

In the teaching process, it is very difficult for students to learn to serve before they are familiar with the feeling of receiving service. At this time, teachers need students to find the space and distance of the ball before they can learn to serve. Scientific training of table tennis as an elective course requires implementing scientific training principles, selecting scientific training contents and methods, and paying attention to monitoring the training process. Table tennis skills and tactics are complex, and each item needs to invest a lot of time and energy in elective courses, so the monitoring of table tennis training in elective courses is a long-term and uninterrupted process. As the main body of monitoring the training process of elective courses, teachers should carefully and scientifically formulate monitoring plans, scientifically select monitoring methods, scientifically implement monitoring processes, and scientifically analyze monitoring results. When playing table tennis, eyes must keep a close eye on the fast coming ball which shuttles back and forth, moves far and near, and rotates constantly so that the eyeball keeps running. Table tennis, as an endurance sport, can make red muscle fibers more than white muscle fibers, improve the types of human muscle fibers, improve eyeball function, and enhance the excitability of the nervous system. Therefore, it can eliminate or alleviate the fatigue of eyes and play a role in preventing myopia.

In teaching, teachers should first let elective courses set up the lofty ideal of climbing the peak of table tennis skills and enhance their motivation to learn and practice. Secondly, we should make the elective courses clear about the specific purpose, requirements, and methods of practice so that they can train well. Finally, various teaching forms should be adopted to keep the elective courses fresh and stimulate their interest in learning.  Figure 1 shows the basic element structure of the integrated service system for physical health of elective courses.

In teaching, teachers should first investigate the table tennis foundation of elective courses and determine their starting height. Secondly, the training system structure of table tennis special sports is shown in Figure 2.

Table tennis coaches also need to pay attention to the guidance of athletes' fighting skills, improve the individual skills of athletes, and reasonably control the practice density and intensity of table tennis. Comparison of muscle contribution rate by different methods is shown in Figure 3.

The effect of table tennis on strengthening muscle speed and strength in elective courses: in table tennis, every movement of the exerciser includes two parts: moving and restoring, and every movement involves many muscle groups. The muscles involved in any movement must undergo two stages: contraction and relaxation. Teachers need to integrate the teaching content so that students can feel the process from easy to difficult and learn easily. In the initial stage of students' technical learning, students are not clear about the concept of correct actions, and they are often prone to wrong actions or redundant actions. We can focus on tracking and photographing students' technical movements so that they can clearly see the situation of completing their movements, find out the shortcomings or mistakes in the movement technology, analyze the reasons, and form the correct concept of movements in their minds. Table tennis exercises with proper intensity through fun and entertainment, which requires thousands of repeated exercises in the practice process, so the muscles have to undergo thousands of exercises. Active contraction and expansion of muscles will greatly increase blood flow in muscles. Teachers should arrange the most suitable exercise load for elective courses according to their physical quality, technical and tactical level, and development potential. Whether it is technical training or tactical training, different training methods should have their own emphasis. Teachers should choose the most suitable training method according to specific training objectives when applying it concretely.

## 4. Conclusions

As a symbol of Chinese sports, table tennis has attracted a large number of elective courses with its unique charm. This paper discusses the influence of table tennis on health. This paper puts forward the reform scheme of teaching plan design of table tennis elective course in colleges and universities, which has a certain reference value for the development of College Physical Education in China. Table tennis training is an elective course; teachers should first implement the scientific training principles, then choose the scientific training contents and methods, and finally pay attention to the monitoring of the training process. In modern society, with the development of science and technology, teachers need to constantly innovate and change teaching methods, so as to effectively improve teaching quality and efficiency and improve students' ability to comprehensively use table tennis special knowledge and skills.

## Figures and Tables

**Figure 1:** The basic element structure of the optional physical fitness and health integrated service system.

**Figure 2:** Table tennis training system structure.

**Figure 3:** Contribution rate comparison.

**Table 1:** Analysis of sampling data of students' physical fitness.

Year	Qualified		Good		Excellent	
	Number of people	Proportion (%)	Number of people	Proportion (%)	Number of people	Proportion (%)
2020	1632	80.1	238	11.7	168	8.2
2019	1621	85.6	245	12.9	28	1.5
2018	1552	79.3	377	19.3	29	1.5

## Data Availability

The data used to support the findings of this study are included within the article.
